# Computed Tomography Image Texture under Feature Extraction Algorithm in the Diagnosis of Effect of Specific Nursing Intervention on Mycoplasma Pneumonia in Children

**DOI:** 10.1155/2021/6059060

**Published:** 2021-10-16

**Authors:** Yuyan Bi, Cuifeng Jiang, Hua Qi, Haiwei Zhou, Lixia Sun

**Affiliations:** ^1^Department of Pediatric Ward, Jinan City People's Hospital, Jinan 271199, Shandong Province, China; ^2^Department of Pediatric Surgery, Jinan City People's Hospital, Jinan 271199, Shandong Province, China; ^3^Department of Nursing, Jinan City People's Hospital, Jinan 271199, Shandong Province, China

## Abstract

To evaluate the effect of specific nursing intervention in children with mycoplasma pneumonia (MP), a feature extraction algorithm based on gray level co-occurrence matrix (GLCM) was proposed and combined with computed tomography (CT) image texture features. Then, 98 children with MP were rolled into the observation group with 49 cases (specific nursing) and the control group with 49 cases (routine nursing). CT images based on feature extraction algorithm of optimized GLCM were used to examine the children before and after nursing intervention, and the recovery of the two groups of children was discussed. The results showed that the proportion of lung texture increase, rope shadow, ground glass shadow, atelectasis, and pleural effusion in the observation group (24.11%, 3.86%, 8.53%, 15.03%, and 3.74%) was significantly lower than that in the control group (28.53%, 10.23%, 13.34%, 21.15%, and 8.13%) after nursing (*P* < 0.05). There were no significant differences in the proportion of small patchy shadows, large patchy consolidation shadows, and bronchiectasis between the observation group and the control group (*P* > 0.05). In the course of nursing intervention, in the observation group, the disappearance time of cough, normal temperature, disappearance time of lung rales, and absorption time of lung shadow (2.15 ± 0.86 days, 4.81 ± 1.14 days, 3.64 ± 0.55 days, and 5.96 ± 0.62 days) were significantly shorter than those in the control group (2.87 ± 0.95 days, 3.95 ± 1.06 days, 4.51 ± 1.02 days, and 8.14 ± 1.35 days) (*P* < 0.05). After nursing intervention, the proportion of satisfaction and total satisfaction in the experimental group (67.08% and 28.66%) was significantly higher than that in the control group (40.21% and 47.39%), while the proportion of dissatisfaction (4.26%) was significantly lower than that in the control group (12.4%) (*P* < 0.05). To sum up, specific nursing intervention was more beneficial to improve the progress of characterization recovery and the overall recovery effect of children with MP relative to conventional nursing. CT image based on feature extraction algorithm of optimized GLCM was of good adoption value in the diagnosis and treatment of MP in children.

## 1. Introduction

Mycoplasma pneumonia (MP) is a common respiratory disease in children. It is caused by mycoplasma pneumoniae infection and is often associated with atelectasis and large lung infiltration. It can cause extrapulmonary multisystem complications [1, 2]. Mycoplasma pneumonia in children is mainly transmitted by respiratory droplets, which then invades the respiratory mucosa. Through its special structure, it is closely adsorbed on the receptor of the cell membrane. It can then multiply and release toxic substances, which can trigger a cascade of symptoms. The prevalence rate of this disease is very high throughout the year, especially in winter. Mycoplasma pneumonia in children generally presents a subacute onset, and the clinical symptoms are usually dry cough, sore throat, headache, and unsteady fever. Sometimes, a severe cough with normal body temperature may be present [3]. If not treated in time, it will bring multisystem and organ damage to the children, and the skin will appear measles-like changes [4]. Specific nursing is a targeted approach to quality care, whose core is people-oriented. It embodies the humanistic spirit and respects the life value, personal dignity, and personal privacy of patients. Patients are greatly helped in rehabilitation treatment by advocating humanized service concept, paying attention to humanized nursing management, and creating humanized service environment [5, 6].

Relevant studies showed that MP is often manifested as the separation of clinical symptoms, signs, and imaging features, and the abnormal rate of pulmonary imaging is substantially higher than the positive rate of pulmonary signs [7]. Clinical examination of MP mainly adopts imaging methods, among which chest X-ray has a high spatial resolution for patient scan. It can reflect the overall condition of the lung, showing interstitial infiltration, lobular, lobular consolidation, and hilar lymph node enlargement. However, due to the overlapping relationship between the front and the rear, the resolution of pulmonary fine lesions is limited to a certain extent, so it is relatively difficult to detect early or ultraearly lesions [8, 9]. High-resolution CT scan can display patients' pulmonary lesions on multiple levels, which is conducive to accurate positioning and clear extent and range of lesions [10, 11]. Feature information extraction is an important work in medical image processing. Different image data need to be processed by different methods, such as the texture feature extraction method based on statistics, the feature extraction method based on frequency, and the feature extraction method based on model [12, 13]. Gray level co-occurrence matrix (GLCM) is the data used to describe the texture related information among image pixels. It can calculate the similarity of gray levels between different pixel points in a specific distance and direction to describe the overall texture information of the image [14] and effectively reduce the time of texture feature calculation and improve the efficiency of the algorithm. Therefore, a novel feature extraction algorithm based on GLCM was proposed and applied to the CT image evaluation of MP in children.

To sum up, the analysis of image texture features is an important work in clinical diagnosis and treatment. Therefore, 98 children with MP were rolled into the observation group with 49 cases (specific nursing) and the control group with 49 cases (routine nursing). CT images based on feature extraction algorithm of optimized GLCM were used to examine the children before and after nursing intervention, and the recovery of the two groups of children was discussed. This research was developed to comprehensively analyze the adoption of CT image texture feature based on GLCM feature extraction algorithm in evaluating the effect of specific nursing intervention in children with MP.

## 2. Materials and Methods

### 2.1. Research Objects

A total of 98 children with MP who were hospitalized in the hospital from June 15, 2019, to April 3, 2021, were selected as the study subjects, including 42 males and 56 females. All the children were divided into the experimental group (49 cases) and the control group (49 cases) according to different nursing plans. This study had been approved by the medical ethics committee of the hospital. The patients and their family members knew about this study and signed the informed consent.

Inclusion criteria: (I) school-age children, (II) children with acute onset, (III) children with fever and respiratory symptoms, (IV) chest X-ray showed patchy infiltrating opacity, (V) children with complete clinical data, and (VI) the family members signed the informed consent.

Exclusion criteria: (I) children unwilling to cooperate with the examination, (II) children with autoimmune diseases, (III) children who had received medical treatment, (IV) children with mixed pulmonary and extrapulmonary infections found by virus examination, and (V) children who quitted the experiment.

### 2.2. Imaging Examination

Philips Brilliance iCT 256-slice spiral extremely fast CT was used to perform high-resolution CT examination of the patient's lungs. The scan range was from the tip of the lung to the diaphragm. The scanning parameters were tube voltage of 120 kV, tube current of 30 mA, and fault of 1-2 mm.

Results judgment was as follows. The distribution, morphological characteristics, and the condition of lung, pleura, and mediastinum were evaluated by professional imaging physicians. The lesion involved sites were left (upper, middle, and lower) and right (upper, middle, and lower) lung field. A mediastinal window scan was also performed to evaluate lymph nodes and pleural cavities, such as pleural effusion. The lung features of HRCT mainly included increased lung texture, cord-like shadow, ground glass shadow, small patchy shadow, large patchy consolidation shadow, atelectasis, bronchiole dilatation, pleural effusion, and hilar mediastinal lymph node enlargement.

### 2.3. Feature Extraction Algorithm Based on Optimized GLCM

The GLCM can calculate the similarity between different pixels at a specific distance and gray level in a specific direction to describe the overall texture information of the image [15]. It is supposed that an image is *Q* and the gray level is *z*; then, the GLCM of the image is *z∗z*. From a pixel point *C* with a gray level of *c* to a pixel point *D* that is *e* pixels away, the corresponding pixel points generated by the two points *C* and *D* are (*c*, *d*). Then, the number of all pixels appearing in the image can constitute the elements of the GLCM. In different directions (0°, 45°, 90°, 135°), the GLCM calculation equation is as follows:

(1) $$\begin{array}{c} F_{0}\left(c,d\right)=\left[u-i=e,v-j=0,f\left(i,j\right)=c,f\left(u,v\right)=d|\left[\left(i,j\right),\left(u,v\right)\in Q\right]\right],\\ F_{45}\left(c,d\right)=\left[u-i=e,v-j=e,f\left(i,j\right)=c,f\left(u,v\right)=d|\left[\left(i,j\right),\left(u,v\right)\in Q\right]\right],\\ F_{90}\left(c,d\right)=\left[u-i=0,v-j=e,f\left(i,j\right)=c,f\left(u,v\right)=d|\left[\left(i,j\right),\left(u,v\right)\in Q\right]\right],\\ F_{135}\left(c,d\right)=\left[u-i=-e,v-j=e,f\left(i,j\right)=c,f\left(u,v\right)=d|\left[\left(i,j\right),\left(u,v\right)\in Q\right]\right], \end{array}$$

where *f*(*i*, *j*)=*c* represents the pixel point with the coordinate (*i*, *j*) in the image and the gray value of *c*, *f*(*u*, *v*)=*d* represents the pixel point with the coordinate (*u*, *v*) in the figure and the gray value of *d*, and *F*_0_(*c*, *d*), *F*_45_(*c*, *d*), *F*_90_(*c*, *d*), and *F*_135_(*c*, *d*) represent the number of pixel pairs appearing in the image at a distance of *e* and in the direction of 0°, 45°, 90°, and 135°, respectively.

Figure 1 graphically shows the specific definitions in the directions of 0°, 45°, 90°, and 135°.

To better understand the calculation method of the GLCM, a binary image with a gray level of 8 and a size of 5 × 4 (Figure 2(a)) is taken as an example.  Figure 2(b) shows that the number of occurrences of the element (1,1) in the 0° direction is 1, the number of occurrences of the element (1,2) is 0, and the number of (1,3) occurrences is 1. By analogy, the GLCM in the 0° direction is finally obtained.  Figure 2(c) shows that the number of occurrences of element (1,1) in the 90° direction is 0, the number of occurrences of element (1,2) is 1, and the number of occurrences of (1,3) is 1. Then, the final GLCM in the 90° direction is obtained.

However, the GLCM has a large amount of data, which is not conducive to the extraction of image features and the classification and recognition of images. Therefore, four statistical indicators of energy (Energy), moment of inertia (Contrast), correlation (Correlation), and entropy (Entropy) were redefined to summarize the characteristic information in the GLCM [16, 17].

Energy reflects the correlation between the distribution of image grayscale and image texture, and the size of the energy is directly proportional to the size of the texture. The larger the value of the moment of inertia, the clearer the image texture. Correlation reflects the correlation of the local pixel distribution of the image. Entropy reflects the texture complexity of the target image. The higher the texture complexity, the higher the entropy value, and vice versa, the lower the entropy.

The equations are as follows:

(2) $$\begin{array}{c} \text{Energy}=\sum_{i}\sum_{j}F{\left(i,j\right)}^{2},\\ \text{Contrast}=\sum_{v=0}^{V_{g1}}v^{2}\sum_{i=1}^{V_{g}}\sum_{j=1}^{V_{g}}F\left(i,j\right),\\ v=\left|i-j\right|,\\ \text{Correlation}=\frac{\left[\sum_{i}\sum_{j}\left(i,j\right)F\left(i,j\right)-\alpha_{x}\alpha_{y}\right]}{\beta_{x}\beta_{y}},\\ \text{Entropy}=\sum_{i=2}^{2V_{g}}\log\left(F\left(i,j\right)\right)*F\left(i,j\right). \end{array}$$

Among them, *P*(*i*, *j*) represents the element value at the coordinate (*i*, *j*) in the GLCM, *i*, *j* ∈ [0, *z*]. *z* represents the gray level of the image. Then, the average value of the four directions of the special parameter is used as the final parameter value:

(3) $$\begin{array}{c} \text{Energy}=\frac{\left({\text{Energy}}_{0}+{\text{Energy}}_{45}+{\text{Energy}}_{90}+{\text{Energy}}_{135}\right)}{4},\\ \text{Contrast}=\frac{\left({\text{Contrast}}_{0}+{\text{Contrast}}_{45}+{\text{Contrast}}_{90}+{\text{Contrast}}_{135}\right)}{4},\\ \text{Correlation}=\frac{\left({\text{Correlation}}_{0}+{\text{Correlation}}_{45}+{\text{Correlation}}_{90}+{\text{Correlation}}_{135}\right)}{4},\\ \text{Entropy}=\frac{\left({\text{Entropy}}_{0}+{\text{Entropy}}_{45}+{\text{Entropy}}_{90}+{\text{Entropy}}_{135}\right)}{4}. \end{array}$$

Eight lung cancer CT images, eight lung benign lesion CT images, and eight healthy adult lung CT images were selected, and the energy, moment of inertia, correlation, and entropy parameters of different types of CT images were calculated. The results were shown in Figure 3. When the feature parameters of the image were calculated by energy, entropy, correlation, and moment of inertia, the features of different types of samples were not obvious. Therefore, although the four parameters can describe the texture information of the image, there was no clear distinction between the feature information of different categories, which misled the image classification work.

To solve these problems, vector fitting [18] is proposed to optimize the GLCM, and the four directions of each feature parameter are vectorized. The vector and modulus of these four vectors are regarded as new feature parameters, and they are expressed as follows:

(4) $$\begin{array}{c} \text{Energy}={\overset{⟶}{\text{Energy}}}_{0}+{\overset{⟶}{\text{Energy}}}_{45}+{\overset{⟶}{\text{Energy}}}_{90}+{\overset{⟶}{\text{Energy}}}_{135},\\ \text{Contrast}={\overset{⟶}{\text{Contrast}}}_{0}+{\overset{⟶}{\text{Contrast}}}_{45}+{\overset{⟶}{\text{Contrast}}}_{90}+{\overset{⟶}{\text{Contrast}}}_{135},\\ \text{Correlation}={\overset{⟶}{\text{Correlation}}}_{0}+{\overset{⟶}{\text{Correlation}}}_{45}+{\overset{⟶}{\text{Correlation}}}_{90}+{\overset{⟶}{\text{Correlation}}}_{135},\\ \text{Entropy}={\overset{⟶}{\text{Entropy}}}_{0}+{\overset{⟶}{\text{Entropy}}}_{45}+{\overset{⟶}{\text{Entropy}}}_{90}+{\overset{⟶}{\text{Entropy}}}_{135}. \end{array}$$

The optimized GLCM is applied to the above different categories of CT images (Figure 4). After the characteristic parameter vector fitting, the information difference of energy value, correlation, moment of inertia, and similarity of different categories of CT images are greatly improved. In general, the improved GLCM parameters based on vector fitting solve the problem that the difference of feature information is not obvious.

### 2.4. Nursing Methods

For the control group, routine treatment of anti-infection, physical cooling, antiasthmatic, sedation, oxygen inhalation, and other nursing treatment was performed. Nursing staff should understand the basic situation of children and the history of allergy through asking the children's parents. Appropriate psychological comfort was made to reduce children's fear of emotion.

Observation group nursing was as follows. (I) Physical sign nursing: the heart rate, respiration, pulse, and so on were observed during admission. If the child's temperature was unstable, it should be measured every two hours, and every five hours when the temperature was stable. For children with high fever, physical cooling and drug intervention can be used, while keeping their skin clean. (II) Psychological care: whether children had negative emotions such as irritability and anxiety were timely observed, and children's treatment compliance should be enhanced through language communication and interaction. At the same time, communicate was made with the families of the children, so did the targeted guidance. (III) Nutrition care: high-protein food was added in the diet of children to ensure adequate nutrition of children. (IV) Environmental care: nurse should pay attention to keep the ward clean and hygienic, fresh air, regular cleaning, and disinfection. (V) Propaganda and nursing: nurse should educate family members about disease prevention and control and conduct propaganda brochures, verbal education, and other methods to popularize knowledge about the disease. Nursing staff should closely observe the vital indicators and clinical signs of the children during treatment to avoid the occurrence of acute sudden symptoms.

### 2.5. Curative Effect Indexes

The improvement of clinical symptoms (the cough disappearance time, the time for returning to normal temperature, the disappearance time of lung rales, and the lung shadow absorption time) was recorded during treatment. The recovery of the two groups of children after half a month of treatment was compared and analyzed. The effects of different nursing interventions are shown in Table 1.

### 2.6. Statistical Analysis

SPSS 19.0 was employed for data statistics and analysis. Mean ± standard deviation ($\bar{x}$ ± *s*) was how measurement data were expressed, and percentage (%) was how count data were expressed. The pairwise comparison was performed by analysis of variance. The difference was statistically considerable with *P* < 0.05.

## 3. Results

### 3.1. Summary of Clinical Manifestations of Children

In Figure 5, the clinical symptoms of 98 children included fever, cough, sore throat, headache, fatigue, wheezing, and kicking sound. The cases of fever, cough, and sore throat were 86, 72, and 59, respectively. The onset time of fever was the earliest (1.24 ± 0.66 days), followed by cough (1.86 ± 1.13 days) and sore throat (1.94 ± 0.58 days). Cough lasted the longest (14.12 ± 3.02 days), followed by fever (8.27 ± 2.85 days).

### 3.2. CT Image of MP

Figure 6 shows chest CT images of a 6-year-old female child with no previous history of hypertension, diabetes, infectious disease, or family history (parents were healthy). Physical examination showed that the child was clear with no deformity of the chest, clear sound on percussion of both lungs, clear breath sound on auscultation of both lungs, no rales were heard, the heart rhythm was uniform, no deformity of the limbs and spine, and the movement was free. CT images showed consolidation of the right upper lobe with air bronchial sign. The lesion distribution was wedge-shaped, ground glass shadow around consolidation, interstitial change, and interlobular interstitial thickening was obvious.

### 3.3. CT Image Characteristics of Two Groups of Children after Nursing Intervention

Figure 7 shows the comparison of CT image features between the two groups after nursing intervention. After nursing, the proportion of increased lung texture, stripe shadow, ground glass shadow, atelectasis, and pleural effusion in the observation group was substantially lower than that in the control group (*P* < 0.05). There was no considerable difference in the proportion of small patchy shadow, large patchy consolidation shadow, and bronchiole dilation between the observation group and the control group (*P* > 0.05).

Figure 8 shows CT images of a 7-year-old male child in the experimental group before and after treatment. Contrast-enhanced CT scan before treatment revealed a distinctly unenhanced low-density area with compartments in the right lung consolidation, marked pleural thickening, and enlarged and uniformly marked lymph nodes behind the anterior tracheal vena cava. After three months of treatment, the review found that the general condition was good, with enlarged anterior mediastinum.

### 3.4. Comparison of Symptom Improvement of Two Groups of Children during Nursing

In Figure 9, the cough disappearance time, the time for returning to normal temperature, the disappearance time of lung rales, and the lung shadow absorption time of the observation group were substantially shorter than those of the control group, and the differences were great (*P* < 0.05).

### 3.5. Comparison of Satisfaction after Nursing Intervention between the Two Groups

Figure 10 shows that the proportion of satisfaction and total satisfaction of children in the experimental group after nursing intervention was substantially higher than that in the control group, and the difference was notable (*P* < 0.05). The proportion of unsatisfied children in the experimental group after nursing intervention was substantially lower than that in the control group, and the difference was great (*P* < 0.05).

## 4. Discussion

Mycoplasma pneumonia is one of the common diseases in children, with a high incidence, which is extremely detrimental to children's physical and mental health development. In addition, due to the particularity of the body structure of children, treatment will bring some difficulties, so it is critical to choose reasonable and effective nursing treatment in clinical practice [19, 20]. Moreover, the infection of mycoplasma pneumoniae has a common antigen with the tissues in the body, so the infection will have a chain reaction with the corresponding tissues. Therefore, it is very necessary to clinically treat the disease and provide care for the disease [21]. According to this particularity, 98 children with MP were divided into 49 cases of the observation group (specific nursing) and 49 cases of the control group (routine nursing). Then, CT images based on the optimized GLCM feature extraction algorithm were used to examine the children before and after nursing intervention, and the recovery of the two groups of children was discussed. The clinical manifestations of the children were summarized, and it was found that the clinical manifestations of the 98 children included fever, cough, sore throat, headache, fatigue, and wheezing. The cases of fever, cough, and sore throat were 86, 72, and 59, respectively. The onset time of fever was the earliest (1.24 ± 0.66 days), and the duration of cough was the longest (14.12 ± 3.02 days).

The CT image characteristics of the two groups of children after nursing intervention were analyzed. It was found that the proportion of increased lung texture, stripe shadow, ground glass shadow, atelectasis, and pleural effusion in the observation group was substantially lower than that in the control group after nursing, and the difference was great (*P* < 0.05). This was similar to the findings of Hata et al. [22], indicating that specific nursing intervention can more effectively promote the recovery of children with MP compared with routine nursing. In addition, there was no considerable difference between the observation group and the control group in the proportion of small patchy shadow, large patchy consolidation shadow, and bronchiole dilation (*P* > 0.05), which was different from the research of Branco et al. [23]. The reason may be that the time of review in this study was relatively short and there was not a considerable difference in long-term outcomes in children. In the process of nursing intervention, the cough disappearance time, the time for returning to normal temperature, the disappearance time of lung rales, and the lung shadow absorption time in the observation group were substantially shorter than those in the control group (*P* < 0.05). It was proved that specific nursing measures for children with MP were conducive to improving the progress of children's characterization recovery [24]. After nursing intervention, the proportion of satisfaction and total satisfaction in the experimental group was substantially higher than that in the control group, while the proportion of dissatisfaction was substantially lower than that in the control group (*P* < 0.05), which indicated that the total nursing effect of specific nursing measures on children was substantially better than that of conventional nursing, which improved the satisfaction of children and their families [25].

## 5. Conclusion

In this study, CT images based on optimized co-occurrence matrix feature extraction algorithm were used to examine 98 children with mycoplasma pneumonia before and after nursing intervention and to explore the rehabilitation of the two groups of children. The results showed that, compared with conventional nursing, specific nursing intervention was beneficial to improve the progress of characterization recovery and the overall recovery effect of children with MP. Therefore, CT image based on feature extraction algorithm of optimized GLCM was of good adoption value in the diagnosis and treatment of MP in children. However, the optimized GLCM feature extraction algorithm designed was not trained and learned enough samples, so it is necessary to do further research on its image processing performance in the future. In conclusion, this study provides data support for clinical nursing intervention in children with MP.

## Figures and Tables

**Figure 1:** Calculation direction of GLCM.

**Figure 2:** Calculation of GLCM: (a) a binary image; (b) a GLCM in the 0° direction; (c) a GLCM in the 90° direction.

**Figure 3:** Energy, moment of inertia, correlation, and entropy parameters of different types of CT images (a–c were CT images of lung cancer, CT of benign lung lesions, and CT of healthy adult lungs, respectively): (a) energy; (b) entropy; (c) moment of inertia; (d) correlation.

**Figure 4:** Energy, moment of inertia, correlation, and entropy parameters of different types of CT images after optimization (a–c were CT images of lung cancer, CT of benign lung lesions, and CT of healthy adult lungs, respectively): (a) energy; (b) entropy; (c) moment of inertia; (d) correlation.

**Figure 5:** Summary of clinical manifestations of children: (a) the number of patients; (b) the time and duration of symptoms.

**Figure 6:** A 6-year-old female child's lung CT image.

**Figure 7:** CT image characteristics of the two groups of children after nursing intervention: (a) increased lung texture, cable-like shadow, ground glass shadow, and small patchy shadow; (b) large sheet consolidation, atelectasis, bronchiectasis, and pleural effusion. *Note.*^*∗*^ indicated considerable difference compared with the observation group (*P* < 0.05).

**Figure 8:** CT images of one child in the experimental group before and after nursing.

**Figure 9:** Comparison of symptoms improvement between the two groups during the nursing process: (a) 1 was the time when cough disappeared, and 2 was the time when body temperature was normal; (b) 3 was the disappearance time of lung rales, and 4 was the absorption time of lung shadows. Note: ^*∗*^ indicated considerable difference compared with the observation group (*P* < 0.05).

**Figure 10:** Comparison of satisfaction between the two groups after nursing intervention: (a) the proportion of satisfied, generally satisfied, and dissatisfied; (b) the proportion of total satisfaction. Note: ^*∗*^ indicated considerable difference compared with the observation group (*P* < 0.05).

**Table 1:** Curative effect indexes of nursing intervention.

Nursing effect	Standard
Satisfied	The child's symptoms improved substantially, and the clinical symptoms were relieved
Generally satisfied	The child's symptoms were slightly improved, and other clinical symptoms were partially relieved
Dissatisfied	The child's symptoms did not improve or worsen

## Data Availability

The data used to support the findings of this study are available from the corresponding author upon request.
